# LncRNA NR2F1‐AS1 regulates hepatocellular carcinoma oxaliplatin resistance by targeting ABCC1 via miR‐363

**DOI:** 10.1111/jcmm.13605

**Published:** 2018-03-30

**Authors:** Hai Huang, Jie Chen, Cheng‐Ming Ding, Xin Jin, Ze‐Ming Jia, Jian Peng

**Affiliations:** ^1^ General Surgery of Xiangya Hospital Central South University Changsha China

**Keywords:** ABCC1, hepatocellular carcinoma, miR‐363, NR2F1‐AS1, oxaliplatin resistant

## Abstract

Emerging evidence has validated the vital role of long non‐coding RNA (lncRNA) in the chemoresistance of cancer treatment. In the present study, we investigate the function of lncRNA NR2F1‐AS1 on oxaliplatin (OXA) resistance of hepatocellular carcinoma (HCC) and discover the underlying molecular mechanism. Results revealed that lncRNA NR2F1‐AS1 was up‐regulated in oxaliplatin‐resistant HCC tissue and cells using microarray analysis and RT‐PCR. Meanwhile, ABCC1 protein was overexpressed in OXA‐resistant HCC cells (Huh7/OXA and HepG2/OXA). In vitro, NR2F1‐AS1 knockdown reduced the invasion, migration, drug‐resistant gene (MDR1, MRP5, LRP1) and IC50 value in Huh7/OXA and HepG2/OXA cells. In vivo, NR2F1‐AS1 knockdown decreased the tumour weight of HCC cells. Bioinformatics tools and luciferase reporter assay confirmed miR‐363 targeted the 3′‐UTR of NR2F1‐AS1 and ABCC1 mRNA, presenting that NR2F1‐AS1 promoted ABCC1 expression through endogenous sponging miR‐363. In summary, results conclude that NR2F1‐AS1 regulates HCC OXA resistance through targeting miR‐363‐ABCC1 pathway, providing a vital theoretic mechanism and therapeutic target for HCC chemoresistance.

## 1 INTRODUCTION

Hepatocellular carcinoma (HCC) is one of the most common malignant tumours, accounting for a significant constituent part of cancer‐related death worldwide with an increase every year.^1^, ^2^ HCC is a rapid growth and invasive tumour and has a tendency for high probability of metastasis and recurrence.^3^ The prognosis of HCC patients is still pessimistic, and the 5‐year survival rate is 30%‐40% in China.^4^ Traditional therapeutic methods for HCC, including surgical resection and chemoradiotherapy, are hard to completely solve the tumour progression.^5^ Fundamentally, the molecular mechanisms for HCC metastasis need to sequentially explore.

Long non‐coding RNA (lncRNA) is one type of the vital epigenetics regulatory mechanism, as well as DNA methylation and genomic imprinting. Emerging evidence has indicated the important role of lncRNA in the multiple cancer tumorigenesis, especially in HCC.^6^, ^7^ For example, lncRNA UBE2CP3 was frequently up‐regulated in HCC samples and promotes hepatocellular carcinoma tumour metastasis via regulating epithelial‐mesenchymal transition and inducing cell invasion and migration.^8^ LncRNA Igf2as was upregulated in HCC cells and tissues and controlled hepatocellular carcinoma progression through the ERK/MAPK signalling pathway.^9^

Oxaliplatin resistance is one of the most vital barriers for HCC chemotherapy. LncRNAs have been proved to modulate the chemotherapy resistance of HCC on molecular level. For example, lncARSR is up‐regulated in HCC and lncARSR overexpression enhances the doxorubicin resistance of HCC cells via modulating PTEN‐PI3K/Akt pathway in vitro and in vivo.^10^

In this study, we measure the expression levels of dysregulated lncRNAs in oxaliplatin‐resistant HCC cells and determine the overexpressed NR2F1‐AS1 in HCC. Our results found that NR2F1‐AS1 regulates hepatocellular carcinoma oxaliplatin resistance by targeting ABCC1 via miR‐363, providing a valuable therapeutic target for HCC tumorigenesis.

## 2 MATERIALS AND METHODS

### 2.1 Clinical samples

All study experimental scheme was conducted in accordance with the commitment of Xiangya Hospital, Central South University. All patients enrolled in this study had written the informed consent before surgery. Totally, 47 cases of oxaliplatin‐resistant HCC patients and oxaliplatin‐sensitive patients who undergo resection operation at Xiangya Hospital, Central South University between October 2012 and December 2016 were recruited in this study. The hepatocellular carcinoma tissues were obtained during surgery and then immediately rapid‐frozen for further use.

### 2.2 HCC cell lines

Human HCC cell lines (Huh7, HepG2) and normal liver cell lines (Lo‐2) were provided by the Chinese Academy of Sciences Cell Bank (Shanghai, China). In a humidified atmosphere with 5% CO_2_, HCC cells were cultured in Dulbecco's modified Eagle's medium (DMEM, Gibco, Grand Island, NY) with 10% foetal bovine serum (FBS, Gibco, Grand Island, NY) at 37°C.

### 2.3 Microarray analysis

Four groups of oxaliplatin‐resistant HCC cells (Huh7/OXA) and matched parental cells were sent for the microarray analysis. Briefly, lncRNA microarray analysis was performed using Affymetrix Human Transcriptome Array 2.0 (HTA 2.0) GeneChips (Affymetrix) after RNA was extracted from cells according to Arraystar's standard protocols. Arraystar Super RNA Labeling Kit (Arraystar, Rockville, MD, United States) was used to label cDNA, and GeneSpringGX software (Agilent Technologies) was performed for quantile normalization.

### 2.4 Quantitative real‐time PCR

Total RNA was extracted from HCC tissues specimens and cells using Trizol reagent (Invitrogen, Carlsbad, Calif, United States). At 260/280 nm, the RNA concentration and purity were measured using a NanoDrop ND‐1000 spectrophotometer (Thermo Fisher Scientific, Waltham, MA, United States). cDNA was reversely transcribed using SuperScript First‐Stand Synthesis system (Invitrogen) from total RNA (2 μg). RT‐PCR was performed using SYBR Premix ExTaq II kit (Takara, Dalian, China) and ABI 7500 PRISM 7500 (Applied Biosystems). The primer sequences used are as follows: NR2F1‐AS1, sense: 5′‐CAGCGGTGCAAACCATGTGC‐3′, anti‐sense: 3′‐GCAAGTTGGCTGAACCAAATG‐5′; miR‐5634, sense: 5′‐GGTCCAGATCTACATGCGT‐3′, anti‐sense: 3′‐CAGTCGTTGCGGGTGAGT‐5′; GAPDH, sense: 5′‐CAGTGCCAGCCTCGTCTAT‐3′, anti‐sense: 3′‐AGGGGCCATCCACAGTCTTC‐5′. Each experiment was performed three times. Relative expression was normalized to GAPDH expression and calculated with the 2^−ΔΔCt^ method.

### 2.5 CCK‐8 assay for chemosensitivity

Cell survival rate and chemosensitivity were determined by using a Cell Counting Kit‐8 (CCK‐8, Dojindo, Japan). Briefly, cells (2 × 10^5^ cells per well) were seeded in 24‐well plates. The proliferation vitality was measured by the absorbance (450 nm). The 50% growth inhibition (IC50) was measured according to the reported literature.^11^

### 2.6 Transwell invasion and migration assay

Transwell assays were performed as described previously.^12^ Briefly, Huh7/OXA and HepG2/OXA cells were seeded in Matrigel‐coated upper chambers with a pore size of 8 μm (50 μL Matrigel, BD Bioscience, United States). Medium without serum 10% FBS was added into the upper chamber, and medium with 10% FBS was added into the lower chambers. For 24‐hour incubation, the migrated and invaded cells on the lower membrane surface were fixed and then stained with 20% Giemsa solution. Five random fields were counted per chamber by using an inverted microscope (Olympus, Japan). Each experiment was repeated three times.

### 2.7 Dual‐luciferase reporter assay

Dual‐luciferase reporter assay was performed as described previously.^13^ Briefly, the RNA sequence of NR2F1‐AS1 and ABCC1 mRNA 3′‐UTR containing the putative binding sites of miR‐363 was inserted into pGL3 (Promega, Madison, WI, United States), generating the pGL3‐NR2F1‐AS1(or ABCC1 mRNA) wild‐type/mutant‐type luciferase reporter vector. HEK‐293T cells (3 × 10^4^) were plated in 24‐well plates and cultured and cotransfected with pGL3 wild‐type/mutant‐type vector (100 ng) and miR‐363 mimics/control or (50 nmol/L) using Lipofectamine 2000 (Invitrogen). The Renilla luciferase gene acted as the standard.

### 2.8 Western blot

Protein samples were extracted using radioimmunoprecipitation assay (RIPA) (Beyotime, Shanghai, China) supplemented with protease inhibitors. Then, protein was separated on SDS‐PAGE gels and transferred to PVDF membranes (Bio‐Rad). PVDF membranes were incubated with primary antibody (anti‐ABCC1, 1:1000 dilution, Abcam) and incubated overnight at 4°C. Then, members were incubated with secondary antibody. Finally, the proteins were visualized with an ECL detection system and quantified using ImageJ software (BD, Franklin Lakes, NJ, United States).

### 2.9 Xenograft nude mice assay

Male nude mice (4‐5 weeks old, twenty mice) were purchased from Animal Care and Use Committee of Xiangya Hospital, Central South University. Animals were fed under sterile‐specific pathogen‐free conditions. About 1 × 10^6^ cells were injected into the subcutaneous of mice. After 3 weeks, the mice were killed using cervical dislocation and tumour weight was measured.

### 2.10 Statistical analysis

Quantitative value of NR2F1‐AS1 expression levels and others was presented as the mean ± SD. Statistical significance was evaluated using multivariate analysis of variance (ANOVA) and Student's *t* test using GraphPad Prism (GraphPad Software, La Jolla, CA, United States). *P* < .05 was considered as statistically significant.

## 3 RESULTS

### 3.1 Microarray analysis profiles revealed that NR2F1‐AS1 was up‐regulated in oxaliplatin‐resistant HCC tissue and cells

To discover the potential dysregulated lncRNAs in oxaliplatin‐resistant HCC tissue, human lncRNA microarray analysis was performed in 4 pairs of oxaliplatin (OXA)‐resistant HCC cells and their parental cells. Heat map showed the representative dysregulated lncRNA with more than fourfold changes, including up‐regulated and down‐regulated lncRNAs (Figure 1A). We noticed a novel identified lncRNA, NR2F1‐AS1, was highly expressed in oxaliplatin‐resistant HCC cells. In 47 pairs of oxaliplatin‐resistant HCC samples, RT‐PCR showed that NR2F1‐AS1 was also significantly up‐regulated compared with matched oxaliplatin‐sensitive samples (Figure 1B). Meanwhile, NR2F1‐AS1 expression levels were similarly highly expressed in oxaliplatin‐resistant HCC cell lines compared with parental cell lines (Figure 1C). Therefore, our study preliminarily affirmed the overexpression of NR2F1‐AS1 in oxaliplatin‐resistant HCC tissue and cell lines.

**Figure 1:** NR2F1‐AS1 was up‐regulated in oxaliplatin‐resistant hepatocellular carcinoma (HCC) tissue and cell lines. A, Heat map shows the representative dysregulated lncRNA with more than fourfold changes. Red symbol presented the high‐expression RNAs. Green symbol presents the low‐expression RNAs. B, NR2F1‐AS1 was up‐regulated in 47 cases of oxaliplatin‐resistant HCC tissue compared with oxaliplatin‐sensitive tissue samples. C, RT‐PCR showed that NR2F1‐AS1 was up‐regulated in human oxaliplatin‐resistant HCC cell lines (Huh7/OXA, HepG2/OXA) compared with parental cell lines. Lo‐2 was the normal liver cells. Data are presented as the mean ± SD. *P < .05, **P < .01 compared to control group

### 3.2 ABCC1 was up‐regulated in oxaliplatin‐resistant cells, and NR2F1‐AS1 knockdown suppressed the oxaliplatin resistance of HCC cells

The survival percentage of HCC cells was measured when treated with increasing concentration of OXA. Results showed that Huh7/OXA and HepG2/OXA cells had higher percentage of survival cells compared with their parental Huh7 and HepG2 cells (Figure 2A). Western blot analysis revealed that ABCC1 protein was significantly up‐regulated in Huh7/OXA and HepG2/OXA compared with their parental Huh7 and HepG2 cells (Figure 2B and C). Interfering oligonucleotides were synthesized and transfected into Huh7/OXA and HepG2/OXA cells to decrease NR2F1‐AS1 expression (Figure 2D). RT‐PCR showed that NR2F1‐AS1 knockdown reduced the mRNA expression levels of drug resistance‐related genes, including MDR1, MRP5, LRP1, compared with control cells (Figure 2E). The 50% inhibitory concentration (IC50) value was measured using CCK‐8 assay. Results showed that in Huh7/OXA and HepG2/OXA cells, the IC50 value of NR2F1‐AS1 knockdown was markedly lower than that of empty control group (Figure 2F and G). In summary, results revealed that NR2F1‐AS1 knockdown suppressed the oxaliplatin resistance of HCC cells. Besides, the drug‐resistant protein ABCC1 was up‐regulated in oxaliplatin‐resistant cells.

**Figure 2:** ABCC1 was up‐regulated in oxaliplatin‐resistant cells and NR2F1‐AS1 knockdown suppressed the oxaliplatin resistance of hepatocellular carcinoma (HCC) cells. A, The survival percentage of oxaliplatin‐resistant HCC cells (Huh7/OXA, HepG2/OXA) and their parental cells when treated with increasing concentration of oxaliplatin (OXA). B, C, Western blot showed the ABCC1 protein expression in oxaliplatin‐resistant HCC cells (Huh7/OXA, HepG2/OXA) and their parental cells. D, Interfering oligonucleotides were synthesized and transfected into Huh7/OXA and HepG2/OXA cells. E, RT‐PCR showed the mRNA expression levels of drug resistance‐related genes, including MDR1, MRP5, LRP1. F, G, The 50% inhibitory concentration (IC50) value was measure in Huh7/OXA and HepG2/OXA cells. si‐1#, 2#, 3# present “siRNA‐targeting NR2F1‐AS1.” Data were expressed as mean ± SD. *P < .05, **P < .01 represents statistically difference

### 3.3 NR2F1‐AS1 knockdown suppressed the migration, invasion and tumour growth of oxaliplatin‐resistant HCC cells in vitro and in vivo

Previous results had revealed that NR2F1‐AS1 knockdown suppressed the oxaliplatin resistance of HCC cells. Subsequently, cellular experiments were performed to verify the role of NR2F1‐AS1 in HCC tumour phenotype. Transwell assay showed that in Huh7/OXA and HepG2/OXA cells, NR2F1‐AS1 knockdown decreased the invasive cell number compared to empty vector‐transfected cells (Figure 3A and B). Moreover, for invasion, NR2F1‐AS1 knockdown decreased the migrative cell number compared to empty vector‐transfected cells (Figure 3C and D). Xenograft nude mice assay showed that NR2F1‐AS1 silencing could significantly reduce the tumour weight of neoplasm in Huh7/OXA and HepG2/OXA cells transfected with NR2F1‐AS1 short hairpin RNA (Figure 3E and F). Overall, results concluded that NR2F1‐AS1 knockdown inhibited the migration, invasion and tumour growth of oxaliplatin‐resistant HCC cells in vitro and in vivo, suggesting the potential tumour‐promoting role of NR2F1‐AS1 in oxaliplatin resistance of HCC.

**Figure 3:** NR2F1‐AS1 knockdown inhibited the migration, invasion and tumour growth of oxaliplatin‐resistant hepatocellular carcinoma (HCC) cells in vitro and in vivo. A, Transwell assay showed the invasive cell number in Huh7/OXA and HepG2/OXA cells transfected with NR2F1‐AS1 siRNA compared to empty vector‐transfected cells. B, Quantitative value of invasive cell number. C, Transwell assay showed the migrative cell number in Huh7/OXA and HepG2/OXA cells transfected with NR2F1‐AS1 siRNA compared to empty vector‐transfected cells. D, Quantitative value of migrative cell number. E, Photographs of xenograft mice and neoplasm. F, Tumour weight of neoplasm in mice injected with sh‐NR2F1‐AS1 or empty vector. Data were expressed as mean ± SD. *P < .05, **P < .01 represent the statistical difference

### 3.4 NR2F1‐AS1 sponged miR‐363 with complementary binding at 3′‐UTR

The role of NR2F1‐AS1 in oxaliplatin‐resistant HCC cells had been illustrated in previous experiments. To investigate the potential molecular mechanism of NR2F1‐AS1, bioinformatics prediction tools^14^ (StarBase V 2.0, http://starbase.sysu.edu.cn/mirLncRNA) were performed. Results revealed that miR‐363 shared complementary bound at 3′‐untranslated regions (3′‐UTR) of NR2F1‐AS1 by binding sites (Figure 4A). Luciferase reporter gene assay showed that the luciferase activity was decreased in the combination of NR2F1‐AS1 wild type and miR‐363 mimics (Figure 4B). RT‐PCR showed that miR‐363 expression levels were down‐regulated in oxaliplatin‐resistant HCC cell lines compared with parental cell lines (Figure 4C). Meanwhile, miR‐363 expression was increased in Huh7/OXA and HepG2/OXA cells transfected with NR2F1‐AS1 siRNA compared to empty vector‐transfected cells (Figure 4D). In 15 pairs of oxaliplatin‐resistant HCC samples, RT‐PCR showed that miR‐363 was significantly down‐regulated in oxaliplatin‐resistant samples compared with oxaliplatin‐sensitive samples (Figure 4E). Therefore, above results revealed that NR2F1‐AS1 sponged miR‐363 at 3′‐UTR, indicating the inverse correlation within NR2F1‐AS1 and miR‐363.

**Figure 4:** NR2F1‐AS1 sponged miR‐363 with complementary binding at 3′‐UTR. A, Schematic diagram demonstrated the complementary bound within miR‐363 and NR2F1‐AS1 3′‐UTR with binding sites predicted by bioinformatics programs (StarBase V 2.0, http://starbase.sysu.edu.cn/mirLncRNA). B, Luciferase reporter gene assay was performed in HEK‐293T cells transfected with NR2F1‐AS1 wild/mutant type and miR‐363 mimics/control. C, miR‐363 expression levels were measured in oxaliplatin‐resistant cell lines and parental cell lines using RT‐PCR. D, RT‐PCR showed the miR‐363 expression levels in Huh7/OXA and HepG2/OXA cells transfected with NR2F1‐AS1 siRNA or empty vector. E, miR‐363 was measured in 15 pairs of oxaliplatin‐resistant hepatocellular carcinoma (HCC) samples and oxaliplatin‐sensitive samples. Data were expressed as mean ± SD. *P < .05 represents the statistical difference

### 3.5 NR2F1‐AS1 modulated ABCC1 protein expression through targeting miR‐363

Both NR2F1‐AS1 and ABCC1 were up‐regulated in oxaliplatin‐resistant HCC cells; besides, miR‐363 targeted the 3′‐UTR of NR2F1‐AS1. Next, bioinformatics tools were performed and results showed that miR‐363 shared complementary binding sites with ABCC1 mRNA 3′‐UTR (Figure 5A). Luciferase reporter assay showed that the luciferase activity was decreased when cotransfected with miR‐363 mimics and ABCC1 mild type, suggesting the molecular bond within miR‐363 and ABCC1 mRNA 3′‐UTR (Figure 5B). In Huh7/OXA cells, ABCC1 mRNA expression level was decreased when transfected with miR‐363 inhibitor (Figure 5C). Western blot revealed that NR2F1‐AS1 knockdown decreased the ABCC1 protein expression and miR‐363 inhibitor transfection increased ABCC1 protein expression (Figure 5D and E). Overall, results indicated that ABCC1 acted as the target protein of miR‐363, suggesting the regulation of NR2F1‐AS1 on ABCC1 through targeting miR‐363.

**Figure 5:** NR2F1‐AS1 modulated ABCC1 protein expression through targeting miR‐363. A, Schematic diagram shows the binding sites within miR‐363 and ABCC1 mRNA 3′‐UTR. B, Luciferase reporter assay shows the molecular bond within miR‐363 and ABCC1 mRNA 3′‐UTR. C, RT‐PCR shows the ABCC1 mRNA expression levels in Huh7/OXA cells transfected with miR‐363 inhibitor. D, Western blot images of ABCC1. E, Quantitative ABCC1 protein expression in Huh7/OXA cells transfected with blank vector, miR‐363 inhibitor and/or si‐NR2F1‐AS1. Data were expressed as mean ± SD. *P < .05, **P < .01 represent the statistically difference

## 4 DISCUSSION

Hepatocellular carcinoma is an aggressive malignant tumour with the high recurrence rate.^15^, ^16^ The clinical therapeutic effects of conventional methods are always unsatisfactory.^17^ One of the most vital pathogen is chemoresistance of HCC cells against series of chemotherapeutic drug, including cisplatin, doxorubicin, oxaliplatin.^18^ In the present study, our research team cultures the oxaliplatin‐resistant HCC cells and investigate the role of NR2F1‐AS1 in oxaliplatin resistance.

Long non‐coding RNA (lncRNA) has been wildly verified to participate in the HCC tumorigenesis regulation; simultaneously, lncRNA modulates the chemoresistance of HCC cells.^19^, ^20^ In the present study, we performed lncRNA microarray analysis in OXA‐resistant HCC cells and their parental cells. Moreover, RT‐PCR showed that NR2F1‐AS1 was significantly up‐regulated in 47 pairs of oxaliplatin‐resistant HCC samples compared with oxaliplatin‐sensitive samples, and in oxaliplatin‐resistant HCC cells (Huh7/OXA, HepG2/OXA). The dysregulated expression of lncRNA provides a valuable clue for the discovery of functional molecular that modulates chemotherapy resistance.^21^ For chemoresistance of HCC, lncRNAs regulate the chemosensitivity of HCC corresponding to clinical chemotherapeutic drugs.^10^, ^22^ For example, lncRNA HULC has been reported to be positively correlated with that of Sirt1 protein in human HCC tissues, stabilizing Sirt1 protein and triggering the autophagy to attenuate the chemosensitivity of HCC cells.^23^

In oxaliplatin‐resistant HCC cells (Huh7/OXA and HepG2/OXA), NR2F1‐AS1 knockdown reduces the mRNA expression levels of drug resistance‐related genes, including MDR1, MRP5, LRP1, which indicate that NR2F1‐AS1 silencing could decrease the oxaliplatin resistance. Meanwhile, the IC50 value of NR2F1‐AS1 knockdown was markedly lower than that of empty control group. With the same of NR2F1‐AS1, ABCC1 protein is up‐regulated in the oxaliplatin‐resistant HCC cells. ABCC1 is one of the known multiple drug resistance‐related protein, acting as an effective indicator for the chemotherapy resistance of clinical treatment.^24^, ^25^ Our results showed that both NR2F1‐AS1 and ABCC1 are up‐regulated in these cultured oxaliplatin‐resistant HCC cells. Therefore, ABCC1 might function as a direct function protein of NR2F1‐AS1 to regulate the oxaliplatin resistance.

Bioinformatics prediction tools are an emerging assistant method to help researchers discover the underlying molecular mechanism within lncRNA and protein mRNA.^26^ By means of these online tools (starBase, TargetScan, miRBase), we found that miR‐363 targeted NR2F1‐AS1 3′‐UTR with complementary binding sites. Besides, the expression levels of NR2F1‐AS1 and miR‐363 are inverse, indicating the antagonistic function and enrichment. Fortunately, miR‐363 also targeted ABCC1 mRNA 3′‐UTR. Thus, we assumed that NR2F1‐AS1 modulates the oxaliplatin resistance of HCC cells by targeting ABCC1 protein via sponging miR‐363. Increasing evidence has illustrated the important role of lncRNA in cancer drug resistance via acting as miRNA “sponge.” For instance, lncRNA NEAT1 up‐regulated in renal cell carcinoma tissue and NEAT1 knockdown increase the sensitivity of RCC cells to sorafenib by acting as a competitive sponge for miR‐34a through the miR‐34a/c‐Met axis.^27^

In summary, our study and data investigate the lncRNA expression profiles in oxaliplatin‐resistant HCC cells and determine the role of lncRNA NR2F1‐AS1 in HCC oxaliplatin resistance. Further experiments reveal the regulatory mechanism of NR2F1‐AS1/miR‐363/ABCC1 pathway on HCC oxaliplatin resistance, suggesting the vital role of NR2F1‐AS1 in HCC research and providing the novel therapeutic target.

## CONFLICT OF INTEREST

All authors declare no conflicts of interest.
